# Nursing Process Design of Intravenous Thrombolysis in Elderly Patients with Acute Cerebral Infarction

This article has been retracted.

**DOI:** 10.1155/2022/2047948

**Published:** 2022-07-30

**Authors:** Yuanyuan Xia, Yuan Chen, Rucui Xia, Yunyun Chen, Qian Gu, Qing Lu

**Affiliations:** ^1^Emergency Medicine Department, Zhongda Hospital Southeast University, Nanjing 210000, Jiangsu, China; ^2^Neurology, Zhongda Hospital Southeast University, Nanjing 210000, Jiangsu, China; ^3^Anorectal, Zhongda Hospital Southeast University, Nanjing 210000, Jiangsu, China; ^4^Neurosurgery, Zhongda Hospital Southeast University, Nanjing 210000, Jiangsu, China

## Abstract

The economy of contemporary society is developing rapidly and the society is making continuous progress. The population is aging and diet structure is also adjusted. Acute cerebral infarction(ACI) in the elderly has become a common disease that seriously threatens the health of the elderly. Therefore, research on nursing of senile ACI is of great significance. Nursing is essential in the thrombolytic therapy of cerebral infarction. This article aims to study the process design of intravenous thrombolytic nursing for elderly patients with ACI and the conclusions are as follows: the nursing process has a good nursing effect. This increased the Barthel index of elderly patients with ACI after intravenous thrombolysis care by 15.8 compared with that before care. Compared with the traditional nursing mode, the nursing course and cost are significantly reduced.

## 1. Introduction

Elderly ACI is a disorder of cerebral blood circulation caused by various reasons. It will appear a clinical syndrome of corresponding neurological loss, which is a kind of ischemic stroke. The people who are prone to ACI are mainly middle-aged and elderly people over 50 years old, especially those with basic cardiovascular and cerebrovascular diseases. The main symptoms are headache, dizziness, nausea, vomiting, hemiplegia, weakness, aphasia, choking after drinking water, etc. Depending on the location of the infarction, the specific symptoms and signs will also vary, which may make some patients disabled and lose their labor force, making life inconvenient. But through reasonable treatment and rehabilitation training, most patients can recover or basically recover. But many patients have also lost their lives because of the disease. Especially for the elderly, ACI is a very dangerous disease. At present, the main treatment method for ACI is intravenous thrombolysis. A complete set of efficient nursing process can effectively promote the intravenous thrombolysis treatment of cerebral infarction diseases. Therefore, this paper mainly studies the nursing process design of intravenous thrombolysis in elderly patients with ACI. Early implementation of thrombolytic therapy for acute cerebral infarction patients who meet the indications for thrombolysis can greatly reduce the disability rate caused by cerebral infarction and further improve the level of social labor resources in China.

The innovations of this paper are as follows: (1) based on clinical nursing path design and medical data mining algorithm, it designs a set of intravenous thrombolysis nursing process for elderly patients with ACI. (2) Based on the designed intravenous thrombolysis nursing process for the elderly with ACI, a nursing experiment in the control group and the experimental group was carried out on 90 selected elderly patients with ACI from January 2020 to December 2021. It draws valid experimental conclusions. Because the intravenous thrombolytic therapy for ultra-early cerebral infarction is simple and easy to implement, the drug price is moderate, safe, and reliable, and it is not restricted by factors such as technology, personnel, and equipment.

## 2. Related Work

In recent years, there have been many studies related to ACI in the medical research community. Among them, Fan et al. research aimed to explore the degree of correlation between CYP2C19 gene polymorphisms and ACI in the elderly. He used gene chip technology to detect gene polymorphisms in 72 elderly patients with ACI [1]. Division mainly studied the clinical process of different elderly patients with ACI. He found that cerebral atrophy can buffer the intracranial pressure of cerebral infarction [2]. Bong et al. mainly studied the role of blood perfusion in ACI. He observed 36 ACI patients with blood perfusion therapy. It was found that blood perfusion has a certain therapeutic effect on cerebral infarction [3]. Dong et al. found through experimental studies that serum resistin levels are associated with an increased risk of ACI [4]. Zhai et al. study mainly explored the predictive value of the ratio of neutrophils and lymphocytes to the prognosis of patients with ACI [5]. Zhu et al. aimed to evaluate the activity of antioxidant stress markers in ACI disease. It was found that serum cholesterol and oxidative stress parameters were significantly higher in patients with ACI [6]. However, the experimental procedures of these studies are mostly complicated and the practicality of the research conclusions obtained is not strong enough.

## 3. Nursing Method of Intravenous Thrombolysis in Elderly Patients with ACI

### 3.1. Intravenous Thrombolytic Therapy

Intravenous thrombolytic therapy for elderly patients with ACI refers to the administration of thrombolytic drugs through the intravenous channel of patients within 3 hours after cerebral infarction to dissolve the thrombus and recanalize the occluded blood vessels. Thereby, the blood circulation can be rebuilt as soon as possible, the infarct size can be reduced, and the prognosis can be improved. Intravenous thrombolysis is an important method for the treatment of venous occlusion in ACI. There are two main types of intravenous thrombolysis. The first is peripheral intravenous thrombolysis, that is, thrombolytic drugs such as urokinase, streptokinase, and It-PA are pumped into the peripheral vein. The effect of this thrombolysis is relatively poor, relatively simple, and relatively high in safety. The second method of thrombolysis is to perform catheter-contact thrombolysis by implanting a thrombolytic catheter under interventional surgery. This type of thrombolytic technique is relatively difficult and expensive, but the thrombolytic effect is relatively good. Thrombolytic drugs can come into direct contact with the thrombus, but also have a relatively low risk of bleeding [7, 8]. The schematic diagram of intravenous thrombolysis treatment is shown in Figure 1.

The main links of intravenous thrombolytic therapy include doctor consultation, team visit, CT examination, and medication [9]. According to international guidelines, the recommended duration of each link of intravenous thrombolysis is shown in Table 1.

### 3.2. Clinical Nursing Pathway

A clinical care pathway is the mode of care for a specific clinical disease that a patient receives during a hospital stay. It also refers to a complete set of hospitalization time in the order of hospitalization, which is formulated for specific patient groups, integrating admission guidance and evaluation, various index inspections, medication guidance, basic nursing, health education, psychological care, and discharge guidance. It is a standardized approach to care that integrates holistic care, quality assurance, and continuous improvement. The clinical care pathway is a synthesis of the physician's routine care plan for each patient diagnosis. It can guide nurses to work predictably and proactively. At the same time, it also enables patients to clarify their own nursing and treatment goals, so as to consciously and actively participate in their own disease nursing process and improve the efficiency of disease treatment. It is a disease care management that optimizes, simplifies, and increases efficiency. As a standardized nursing treatment mode, it can greatly shorten the length of hospital stay and control the cost of hospitalization and effectively improve the level of medical care. It is a new nursing model of comprehensive “managed care” that conforms to the cost-benefit law [10, 11]. The clinical nursing technology architecture and implementation are shown in Figure 2.

The clinical care pathway has the following characteristics:

1. Personalization: the clinical nursing pathway provides very detailed planning and guidance for nursing work, but nurses should master its flexibility in the application process. According to the specific conditions of different patients, the path plan can be modified at any time to meet different situations, so as to fully realize the role of the path [12].
2. Timeliness: nursing paths for different diseases have different time limits. In the process of implementing the clinical nursing pathway, it is necessary to follow the sequence plan formulated by the pathway and carry out appropriate nursing measures in a specific time period [13].
3. Coordination: the clinical care pathway is developed by all members of the medical care provider to develop the treatment content and implementation time. It is integrated with nursing, medical, and other personnel. In the nursing process, it is necessary to ensure the integrity of the path, requiring the patient to be the center, nurses, doctors, and other medical personnel to cooperate and communicate with each other, carry forward the team, and serve patients together [14].
4. Effectiveness: a clinical care pathway is a pre-established standard of care. During the implementation process, attention should be paid to the practicality of implementation and strict implementation. Nurses can carry out nursing work in a planned and purposeful manner, and patients can also understand the treatment plan, so that they can actively participate in the nursing process [15].

The clinical care path process is shown in Figure 3.

### 3.3. Medical Data Mining Algorithms

Data mining refers to the process of knowledge discovery and application that extracts unknown and valuable knowledge in the form of rules, patterns, and other forms of knowledge from a large number of noisy data sources without explicit assumptions and uses discovered knowledge to help explain current behavior or predict future outcomes. This technology is more and more widely used under the background of “information explosion and lack of knowledge.” Medical data mining algorithm refers to the mining algorithm for massive medical data [16]. The typical data mining operation steps are shown in Figure 4.

Commonly used medical data mining algorithms include decision tree algorithm and support vector machine algorithm.

#### 3.3.1. Decision Tree Algorithm

Decision tree algorithm is one of the commonly used classical data mining algorithms. The core idea of the decision tree algorithm is to effectively dig and classify some data sets. The information entropy Ent(*S*) is as follows:

(1) $$\begin{array}{c} \text{Ent}\left(s\right)=-\sum_{i=0}^{k}c_{i}s\;\log\;P. \end{array}$$

The information entropy Ent(*A*, *T*, *S*) is as follows:

(2) $$\begin{array}{c} \text{Ent}\left(A,T,S\right)=\frac{\left|S_{i}\right|}{s}\text{Ent }S. \end{array}$$

The information gain is as follows:

(3) $$\begin{array}{c} \text{Gains}\left(A,T,S\right)=\text{Ent}\left(s\right)-\text{Ent}\left(A,T,S\right). \end{array}$$

The principle of the decision tree algorithm is shown in Figure 5.

#### 3.3.2. Support Vector Machine Algorithm

Data mining algorithms are starting from the data of the sample and looking for the data to see the pattern in a very traditional way. The basic idea of the support vector machine algorithm is to achieve the purpose of data mining and classification by processing the data classification interval.

During the operation of the support vector machine algorithm, it first sets the linear characteristic function *g*(*x*) of the following general form:

(4) $$\begin{array}{c} g\left(x\right)=w*x+b. \end{array}$$

Then, the linear classification equation that needs to be constructed for the data sample points can be defined as follows:

(5) $$\begin{array}{c} f\left(x\right)=w\left(x+b\right). \end{array}$$

At the same time, the expression for the data classification interval is as follows:

(6) $$\begin{array}{c} \text{margin}=\frac{2}{\left\|w\right\|}. \end{array}$$

To maximize the value of this classification interval, it can be converted into equivalent at the same time, so that ‖*w*‖ is the smallest, that is, as follows:

(7) $$\begin{array}{c} y_{i}=\left(w*x\right)+b-1, \end{array}$$

and *y*_*i*_ ≥ 0. To sum up, in order to make the classification interval margin complete the equivalent replacement, it is necessary to correctly divide all the sample points. After the correct classification is made in this way, the sample data training points need to meet the following constraints:

(8) $$\begin{array}{c} \sum_{i=1}^{n}y_{i}a=0,\;a\geq 0. \end{array}$$

With the introduction of the above constraints, it is necessary to solve the maximum value of the multiplier of the Lagrange method in the following dual variable:

(9) $$\begin{array}{c} Q\left(a\right)=\sum_{i=1}^{n}a_{i}-\frac{1}{2}\sum_{i,j=1}^{n}a. \end{array}$$

If *a*_*i*_ is the optimal solution obtained by the above function, then

(10) $$\begin{array}{c} w=\sum_{i=1}^{n}ay. \end{array}$$

This shows that the optimal linear combination support vector machine of training sample vectors is the vector set of weight coefficients for optimal classification. It is calculated using the Lagrange function as follows:

First it makes:

(11) $$\begin{array}{c} L\left(w,a,b\right)=\frac{1}{2}\left\|w\right\|-\sum_{i=1}^{i}a_{i}\left(w+b\right)-1. \end{array}$$

Then, there are

(12) $$\begin{array}{c} \frac{\alpha }{\alpha b}L\left(w,b,a\right)=0, \end{array}$$

and

(13) $$\begin{array}{c} \frac{\alpha }{\alpha w}L\left(w,b\right)=a. \end{array}$$

Among them,

(14) $$\begin{array}{c} W\left(a\right)=\sum_{i=1}^{i}\alpha_{i}-\frac{1}{2}a_{i}. \end{array}$$

Then,

(15) $$\begin{array}{c} f\left(x\right)=\mathrm{sgn}\left(\sum_{i=1}^{i}y_{i}\alpha_{i}+b\right). \end{array}$$

The optimal classification function of the support vector obtained after solving the above problem is as follows:

(16) $$\begin{array}{c} f\left(x\right)=\mathrm{sgn}\left(w*x+b\right)a_{i}y_{i}. \end{array}$$

## 4. Design Experiment of Intravenous Thrombolysis Nursing Process for Elderly Patients with ACI

### 4.1. Experimental Design

The main methods and procedures of this experiment of intravenous thrombolysis nursing process design for elderly patients with ACI are as follows: first, it uses random sampling to select 90 elderly ACI cases from January 2020 to December 2021 as the experimental subjects of this experiment. The 90 elderly patients with ACI were divided into control group and experimental group. Among them, there were 40 people in the control group and 50 people in the experimental group. The patients in the experimental group were treated with a pre-established intravenous thrombolysis nursing model based on clinical nursing paths and medical data mining algorithms. After the end of the nursing process, the changes in Barthel index and changes in length of stay and costs at discharge were compared between the two groups. Through this, it can judge the feasibility and effect of intravenous thrombolysis nursing process for elderly patients with ACI based on clinical nursing path in the rehabilitation nursing of elderly patients with ACI.

The basic data of the control group and the experimental group in this experiment are shown in Table 2.

In this experiment, the pre-established nursing process is as follows: on the 1st and 2nd day of admission, the patient's condition is mainly fully understood. Then, it determines specific rehabilitation care methods, and correctly implements the doctor's orders to ensure that basic care is in place. On the 3rd to 7th day, it further improves the relevant inspections, and carries out corresponding drug guidance and psychological care. Patients at this stage begin to perform 15–30 minutes of heavy-to-light exercise 2-3 times a day. In the second week, the nurses assist the patients to conduct re-examination CT and other related examinations, and at the same time strengthen the basic nursing care, diet, and medication guidance for the patients. At this stage, patients can also be taught to do some active rehabilitation exercises according to the actual situation. In the third week, according to the patient's condition, the corresponding functional training and daily life ability training will be given and the patient will be taught some rehabilitation methods for the affected limb. In the 4th week, it is necessary to explain the results of various re-examinations to the patients and their families, and at the same time to further improve the basic nursing care, instruct the patients to follow the doctor's orders and give drug guidance. At the time of discharge, the patient needs to be given the necessary discharge guidance. For example, the patients should be instructed to pay attention to the precautions in all aspects of daily life after discharge from the hospital, the blood pressure of the patients should be measured, the nursing treatment effect should be consolidated, and the patient's disease recurrence should be prevented as much as possible.

The above is the whole process of intravenous thrombolytic nursing for elderly patients with ACI designed for this experiment. Next, this experiment will carry out nursing treatment for the patients in the experimental group according to this nursing process. At the same time, patients in the control group were treated according to the traditional nursing model.

### 4.2. Barthel Index Test and Comparison

After the end of care for both groups of patients, the experiment will first test the Barthel index of the two groups of patients at the time of discharge according to the actual nursing and treatment results and compare it with the Barthel index at the time of admission. The test and comparison results of the Barthel index of the two groups of patients at the time of admission and discharge are shown in Figures 6 and 7

Combining Figures 6 and 7, the Barthel index of the control group changed from 35.6 at admission to 45 at discharge. The Barthel index of the experimental group changed from 36.8 at admission to 52 at discharge. According to international standards, the higher the Barthel index value, the better the nursing effect. In contrast, the Barthel index of the experimental group increased significantly, and the Barthel index at discharge was 7 higher than that of the control group using the traditional care model. This preliminarily shows that the nursing process of intravenous thrombolysis for elderly patients with ACI based on clinical nursing path and medical data mining algorithm designed in this paper has better nursing effect than traditional nursing process.

### 4.3. Statistics and Comparison of Hospitalization Days and Expenses

Finally, the statistical results of the number of days of hospitalization and hospitalization fees for the experimental group and the control group in this nursing process are shown in Figure 8.

As can be seen from Figure 8, the total hospitalization days of the patients in the control group were 20 days and the total hospitalization cost was 15,000 yuan. The total length of stay in the experimental group was 15 days, and the total hospitalization cost was 12,000 yuan. Obviously, the total hospitalization days of the patients in the experimental group were 5 days less than that of the patients in the control group and the corresponding total hospitalization expenses were also reduced by 3,000 yuan. This side shows that the intravenous thrombolysis nursing process for elderly patients with ACI based on clinical nursing path and medical data mining algorithm designed in this paper has better nursing effect. This makes the treatment duration and cost of patients in the experimental group lower than those in the control group using the traditional care model.

To sum up, the conclusion was drawn from the experiment of intravenous thrombolytic nursing process design for elderly patients with ACI. Compared with the traditional nursing process, the nursing process of intravenous thrombolysis for elderly patients with ACI based on clinical nursing path and medical data mining algorithm designed in this paper has more obvious nursing effect. This reduces the duration and cost of intravenous thrombolytic nursing for elderly patients with ACI, and the patient's Barthel index also increased by 15.8 compared with before nursing.

## 5. Discussion

Elderly ACI is a cerebrovascular disease that seriously endangers the life of elderly patients, with a very high fatality rate. Therefore, both doctors and ordinary people in contemporary society are paying more and more attention to the disease. In the treatment of ACI in the elderly, intravenous thrombolysis is the main treatment method. In the process of intravenous thrombolytic therapy for ACI in the elderly, proper nursing process is one of the indispensable conditions for curing the disease.

## 6. Conclusions

The design of the nursing process of intravenous thrombolysis in elderly patients with ACI is of great significance for the treatment of elderly patients with ACI. This paper draws conclusions on the nursing process design of intravenous thrombolytic therapy for elderly patients with ACI. Compared with the traditional nursing process of intravenous thrombolysis for elderly ACI, the nursing process based on clinical nursing path and medical data mining algorithm has better nursing effect. This increased the Barthel index of the elderly patients with ACI at discharge by 15.8 compared with that before nursing, and their hospitalization and total hospitalization costs were lower than those of patients using traditional care models. This conclusion fully shows that the nursing process of intravenous thrombolytic therapy for elderly patients with ACI based on clinical nursing path and medical data mining algorithm design has considerable nursing effect of intravenous thrombolytic therapy for elderly patients with ACI. However, in view of the limitations of the research conditions and research level, the research in this paper also has some shortcomings in some aspects, and it is hoped that it can be improved in future research. It is also believed that there will be more research related to the nursing process design of intravenous thrombolytic therapy for elderly ACI diseases in the future, so as to continuously promote the development of medical technology for the treatment of elderly ACI diseases. Although intravenous thrombolytic therapy for acute cerebral infarction has many defects and deficiencies in its vascular recanalization rate and reocclusion rate, because of its simplicity, rapidity, and noninvasiveness, it is not suitable for arterial thrombolysis and mechanical thrombectomy. It is still an effective treatment method in grass-roots hospitals, which is worthy of promotion in grass-roots medical institutions. However, there is still a lack of large-scale evidence-based medical data support for combined thrombolysis, the technical support requirements for personnel setting are high, and the treatment cost is relatively expensive, which limits further clinical promotion and use.

## Figures and Tables

**Figure 1:** Schematic diagram of intravenous thrombolytic therapy.

**Figure 2:** Clinical nursing technology architecture and Implementation. (a) Technical architecture. (b) Implementation.

**Figure 3:** Clinical care pathway flow.

**Figure 4:** Data mining steps.

**Figure 5:** Principle of decision tree algorithm.

**Figure 6:** Barthel index of control and experimental groups at admission. (a) Barthel index of control group at admission. (b) Barthel index of experimental group at admission.

**Figure 7:** Barthel index of experimental group and control group at discharge. (a) Barthel index of the control group at discharge. (b) Barthel index of the experimental group at discharge.

**Figure 8:** Days of hospitalization and total hospitalization costs in the control and experimental groups. (a) Number of days in hospital. (b) Total cost of hospitalization.

**Table 1:** Recommended duration of each link of intravenous thrombolysis.

All aspects of intravenous thrombolysis	International guideline recommended duration (minutes)
Doctor admissions	≤10
CT examination	≤15
CT report acquisition	≤25
Intravenous thrombolytic drugs	≤45

**Table 2:** Basic information on admission to the control group and the experimental group.

Feature	Control group	Test group	Value of *P*
Number of cases	40	50	0
Age	72–81	70–83	0.66
TACI, *n* (%)	5 (4.8)	4 (3.1)	0.96
PACI, *n* (%)	30 (18.0)	34 (28.0)	0.97

## Data Availability

No data were used to support this study.
